The article "Government-Enterprise Collusion and the Effectiveness of Environmental Regulations: Implications for Public Health" was published in 2023. Journal: J Environ Public Health.

# Government-Enterprise Collusion and the Effectiveness of Environmental Regulations: Implications for Public Health

**DOI:** 10.1155/2023/3958944

**Published:** 2023-02-09

**Authors:** Shuang Zhao, Lin Peng, Haiyan Zhou, Feng Hu

**Affiliations:** ^1^Business School, Hohai University, Nanjing 211106, China; ^2^School of Economics and Management, Chuzhou University, Chuzhou 239000, China; ^3^Institute of Digital Economy and Green Development, Chifeng University, Chifeng 024000, China; ^4^Global Value Chain Research Center, Zhejiang Gongshang University, Hangzhou 310018, China

## Abstract

Effective environmental management will create a win-win situation for building an ecological civilization with the potential to control the COVID-19 pandemic. From the perspective of government-enterprise collusion (GEC), this study analyzes the moderating effects of the officials' promotion incentives and turnover on the effectiveness of environmental regulations utilizing a panel dataset on 276 cities in China from 2003 to 2019. The study reveals the following empirical results: First, promotion incentives positively moderate the relationship between environmental regulations and environmental pollution, mainly air pollution; results for water pollution are not significant. Compared with general cities, the positive moderating effect of promotion incentives in high-level cities is weaker and the negative moderating effect is more potent. Additionally, the moderating effect of promotion incentives is predominantly positive in the new developmental stage from 2013 to 2019. Second, the negative moderating effect of officials' turnover on the effectiveness of environmental regulations is mainly observed for water pollution but not evident for air pollution. Compared with high-level cities, officials' turnover in general cities is more conducive to the effectiveness of environmental regulations. These findings provide beneficial insights for promoting green growth by improving official governance and destroying GEC.

## 1. Introduction

COVID-19 poses a severe threat to public health around the world. Governments have taken measures such as travel restrictions and city blockades to deal with the spread of the pandemic. In addition to spatial strategies such as isolation and interdiction, some studies have found that environmental pollution, especially air pollution, significantly impacts the spread of COVID-19 [1–3]. Air pollutants (such as PM_2.5_, PM_10_, NO_2_, and SO_2_) act as carriers to spread the COVID-19 virus and also affect lung health, making those infected more vulnerable to the virus. Therefore, strengthening pollution governance will contribute to alleviating environmental degradation and controlling the COVID-19 pandemic. China has made tremendous economic achievements since it began to open up and reform its economy. However, the ensuing extensive development also brought severe environmental pollution. According to China's 2020 Eco-Environment Bulletin, 43.3% of China's cities (337) exceeded the standard of ambient air quality and 43.6% of the 10,242 groundwater quality monitoring points registered Class V water. Governments at all levels have strengthened the enforcement of environmental regulations; nevertheless, the actual results are not promising [4, 5]. The report “Confessions of the Director of the Environmental Protection Bureau: I am the Director of Public Relations Showmanship” sparked public thinking. According to the report, although the concept of green development continues to gain popularity, some regions still maintain the former development model, in spite of high pollution and high emissions, under the wraps of promotional tournaments and dependence on traditional development models. Enterprises contribute to tax revenue, while local governments provide shelter for nonclean production. Environmental damage is still tacitly permitted and tolerated, thus creating high growth and heavy pollution concurrently. Western mainstream economic theories cannot effectively explain China's development model of growth and pollution at high levels simultaneously. Some studies advance the theory of government-enterprise collusion (GEC) to integrate growth and pollution into the same analytical framework [6, 7].

The asymmetrical information between the central and local governments provides favorable conditions for collusion, and the officials' promotion incentives to pursue short-term economic growth are undoubtedly an essential driving factor for GEC [7, 8]. Local officials are desperate to demonstrate their performance and competence during their short-term service under the tenure system, which requires mandatory retirement at a fixed age; conversely, the high turnover rate of local officials affects the stability of the collusion network. Evidence shows that local officials frequently change, and their terms are generally short in China. Between 2007 and 2017, nearly 80% of municipal party secretaries were reassigned in less than five years and more than 20% were in office for less than a year [9]. Frequent turnover of principal local officials undermines the collusion network and creates a deterrent-sensitive period. What are the effects of promotion incentives and officials' turnover rates on environmental regulations in the context of collusion enhancement and deterrence perspectives? Are these effects heterogeneous according to pollutant and city class? The answers to these questions are important to achieve a win-win situation for constructing an ecological civilization and controlling the COVID-19 pandemic.

The marginal contribution of this study is threefold. First, the study probes the moderating effects of promotion incentives and officials' turnover on the relationship between environmental regulations and environmental pollution. To the best of our knowledge, previous research studies focused on the direct effects of promotion incentives and officials' turnover on the environmental system, and few studies examined the moderating effects of both. Our analysis incorporates promotion incentives and officials' turnover into the effectiveness of environmental regulations from the perspective of GEC and reveals the moderating effects of promotion incentives and officials' turnover. Second, the study introduces GEC into the research of environmental regulatory effectiveness, which will expand the application scenario of the theory of GEC and the research perspective of environmental regulatory effectiveness. Previous studies introduced GEC to issues such as high housing prices, food safety, and overcapacity, but few combined GEC and environmental regulatory effectiveness. Based on this research gap, the mechanisms for collusive reinforcement and breaks caused by promotion incentives and officials' turnover are discussed and their moderating effects on the effectiveness of environmental regulations are examined. Finally, our research focuses on pollutant heterogeneity. Unlike the existing literature that focused on a single pollutant or pollution composite index, our study includes multiple pollutants to investigate the performance of strategic emission reduction due to pollutant heterogeneity.

The rest of the study is organized as follows: Section 2 is the literature review.  Section 3 presents the theoretical logic and research hypotheses.  Section 4 includes the introduction to model construction and variable data description, and Section 5 shows the empirical results and analyses. The final section contains the conclusions, policy implications, and limitations of the study.

## 2. Literature Review

Scholars have conducted some research studies on the effectiveness of environmental regulations, which can be divided into two categories according to internal and external research perspectives. The first category concerns the impact of the heterogeneity of environmental regulations on technological innovation and environmental improvement. Environmental regulations can be divided into market-incentive environmental regulations (MERs) and command-controlled environmental regulations (CERs). The former occurs mainly through the environmental protection tax system and emission trading to incentivize each subject to reduce emissions; the latter sets emissions standards and even mandatory shutdowns. The effectiveness of regulations is also quite different due to mechanism and application conditions. Sun et al. [10] found that the incentive effect of MER on innovation in Chinese high-tech enterprises was more significant and that flexible regulatory tools and implementation methods were more conducive to encouraging enterprises to carry out innovative activities. Similarly, Fang and Shao [11] stated that MER promoted regional green technology innovation, while CER inhibited it based on local data in China. However, MER is not always optimal but depends on the heterogeneity of regulated objects. For example, Zhu et al. [12] argued that CER and voluntary regulations positively impacted the green transformation of Chinese steel companies, while MER did not. The second category of studies focuses on the external conditions of environmental policy implementation. Huang and Lei [13] found that the marketization level positively modified the relationship between environmental regulations and enterprises' green investment, which was more significant among nonstate-listed enterprises. Other studies analyzed the fiscal decentralization level, industry differences, and industrial agglomeration [14–16].

Local government officials are an important external factor influencing the effectiveness of environmental regulations in China [17]. Seeking political promotion can be considered the most critical career incentive for Chinese officials [18, 19]. In the context of absolute power held by local governments, the promotion incentives and position turnover of government leaders significantly impact regional economic, social, and environmental systems. Scholars have also conducted research studies on the impact of promotion incentives and officials' turnover on environmental pollution [20–22]. On the whole, there is a consensus that competing for promotions with a one-sided emphasis on economic growth exacerbates environmental pollution. Furthermore, relevant research studies have explored the mechanisms behind the impact of promotion incentives and officials' turnover on environmental pollution, including the perspectives of GEC and anticipatory effects. Yu et al. [23] stated that under China's current official evaluation system, local governments collude with enterprises to achieve economic growth, which may lead to more severe environmental pollution. Song et al. [24] analyzed the effects of the frequency and predictability of officials leaving office in Chinese cities on air quality in their jurisdictions and found that air pollution spiked in the year prior to the leadership turnover when the incumbent anticipated a change of term. Local leaders are keener on short-term policies to stimulate economic activities. They demonstrate their competence to superiors at the expense of air quality when officials' turnover is frequent and predictable. From the perspective of GEC, promotion incentives and officials' turnover can be organically linked, which provides a valuable reference and inspiration for our research.

The existing literature has explored the impact of promotion incentives and officials' turnover on environmental pollution, but there is still room for discussion about the impact of both on environmental systems. Previous research studies focused on the direct effects of promotion incentives and officials' turnover on environmental pollution; however, the moderating effects are not sufficiently explored, and research from the perspective of GEC is even scarcer. Environmental regulations are currently the primary means for governments to strengthen environmental governance. Systematically, exploring the effects of promotion incentives and officials' turnover on the effectiveness of environmental regulations will facilitate the improvement of environmental governance. Meanwhile, it can also provide a reference for clarifying the mechanisms related to official governance and green development. Our study constructs a theoretical logic that promotion incentives and officials' turnover affect the efficiency of environmental regulations from the perspective of GEC and investigates the moderating effects involved. The main work of this study includes the following points: First, based on the perspective of GEC, we analyze the reinforcing and deterring effects of promotion incentives and officials' turnover on GEC to establish the moderating mechanisms of promotion incentives and officials' turnover on the efficacy of environmental regulations. Second, we examine the impact of environmental regulations on environmental improvement by employing city panel data and using it as a benchmark to explore the moderating effects, focusing on the strategic manifestation of collusion arising from pollutant and city-rank heterogeneity. Ultimately, from the empirical research, we draw policy implications to curb GEC and improve the efficiency of environmental governance.

## 3. Theoretical Logic and Research Hypothesis

### 3.1. GEC to Distort Environmental Regulations

The distortion of environmental regulations caused by GEC can be divided into explicit and implicit manifestations. On the one hand, pollution control and green technology research require large amounts of capital investments, which will increase operating costs, reduce corporate profits, and affect the performance of local economic development. To achieve prosperous economic performance in the short term and especially to boost the economy after the COVID-19 pandemic, local governments lower environmental enforcement standards, relax environmental supervision efforts, and even shelter polluting enterprises during inspections by higher level governments. This explicit distortion of environmental regulations by GEC is easy to observe. On the other hand, local governments introduce and develop heavy-polluting industries by lowering environmental requirements, further exacerbating local environmental pressures. The explicit and implicit distortions of environmental regulations by GEC are intertwined, with local officials and enterprises deriving economic performance and operating profits from collusion and regulatory distortions, respectively. Enterprises lose the motivation and incentive to control pollution gradually, and the effectiveness of environmental regulations diminishes significantly.

### 3.2. Promotion Incentives to Establish GEC

The widespread principal-agent relationships between central and local governments inevitably lead to information asymmetry. The degree of information asymmetry is likely to deepen, especially in the context of economic decentralization, which has become one of the critical challenges in the modernization of national governance. Although the central government collects local information through various means, such as the establishment of six regional inspection centers for environmental protection in 2006 to alleviate the information asymmetry dilemma, the effect is still limited compared to the massive amount of information in economic and social systems. GEC is easy to establish in a situation where the central or higher level government does not have complete access to local information.

Asymmetric information prevents the central government from comprehensively understanding all local government behaviors. To avoid moral hazards, the central government has developed different assessment systems for local officials in various stages of development. The bias of assessment systems on the gross domestic product (GDP) and fiscal tax revenue indicators profoundly impacts the degree of GEC. The official appraisal system since 1949 can be roughly divided into three stages (1949–1978, 1978–2002, and 2002–2019). Before China's economic reform and opening up, to consolidate the political order and the needs of a highly centralized planned economy, the main criterion for assessing officials was political loyalty. From the reform era to the beginning of the 21st century, however, economic development became the focus of work, and economic assessment was the principal criterion at this stage. With the 16th Congress of the Communist Party of China (CPC) in 2002 as the node, the officials' appraisal criteria gradually turned to a multidimensional appraisal with comprehensive economic-environmental-social coordination [18]. Although the official evaluation criterion is gradually reversing the drawback of focusing purely on the GDP, local officials still regard economic performance as a bargaining chip for political promotion due to the high visibility of economic indicators and the lagging effect of environmental governance [25, 26]. In particular, unlike the promotion of high-level officials, which is influenced by noneconomic factors such as “nepotism,” “political affiliation,” and “loyalty” [27], the promotion of low-level officials is highly linked to economic performance.

There is a strict retirement policy in China's administrative system: 60 years for prefecture-level municipal officials and 65 for provincial ministerial-level officials. In 1986, the CPC Central Committee put forward the reform of rejuvenating the leadership team. Therefore, the age of officials has become an important consideration for political promotion. Further analysis reveals that the probability of promotion is inversely related to the length of tenure [25] and promotion incentives motivate local officials to attain economic achievements under limited terms. Therefore, this study proposes Hypothesis 1:

H1: In the context of perverse incentive structures and asymmetric information, promotion incentives will positively moderate the relationship between environmental regulations and environmental pollution, which is detrimental to environmental improvement.

### 3.3. Officials' Turnover to Deter GEC

Information asymmetry of multiple dimensions often exists in transition economies. In addition to information asymmetry between the central and local governments, there is also information asymmetry between enterprises and local governments. China's traditional government-enterprise relationship has been characterized by dependency for thousands of years. Under such circumstances, enterprises are always incentivized to establish stable relationships with governments to obtain more resources efficiently. According to the survey of more than 12,000 enterprises in mainland China conducted by the World Bank in 2005, each enterprise spent an average of nearly 60 days a year, dealing with government core departments, and the top 5% of enterprises spent up to 170 days. Although different levels of government have implemented a series of initiatives to streamline administration and delegate powers since 2012, there are still some areas where “time tax” remains high for enterprises. If an official serves in a city long term, collusion is more likely to occur because it is easier to manipulate local regulators [28]. The exchange of officials has been incorporated as a formal system in the officials' governance since 1990. Under the current system, the transfer of officials does not require strict adherence to the tenure of the local leadership team but shows the characteristics of “flexible terms of office and transfers at any time.” Frequent officials' turnover can break the stable collusive relationship [29] and create a politically sensitive period. The deterrent effect and uncertainty will be more substantial, especially when officials fall for corruption. Such collusive shocks and uncertainty can profoundly affect enterprises' behaviors [30, 31]. When corruption is significant in the environmental field, political instability caused by the officials' turnover can positively impact the stringency of environmental regulations. Corruption weakens the seriousness of environmental regulations, but this effect disappears as political instability increases [32]. Therefore, the aforementioned discussion leads to the development of Hypothesis 2 which is as follows.

H2: Officials' turnover has a positive effect on breaking the collusion network, thus forming a politically sensitive period. Pollution will be curbed, and environmental regulations will be enforced. Consequently, officials' turnover will negatively moderate the relationship between environmental regulations and pollution, thereby contributing to environmental improvement.

Utilizing the two aforementioned hypotheses, the logical framework of this study is illustrated in Figure 1.

## 4. Methodology

### 4.1. Variable Selection

#### 4.1.1. Dependent Variables

Pollution emissions are mainly derived from industry, so environmental pollution is measured by three types of pollutants: industrial wastewater emissions, industrial soot emissions, and industrial sulfur dioxide (SO_2_) emissions. These emissions include two dimensions of pollutant emissions per unit of industrial value added (i.e., WaterI, SootI, and SO_2_I) and total pollutant emissions (i.e., water, soot, and SO_2_).

#### 4.1.2. Independent Variable

Environmental regulation (ER) is the independent variable of this study. There is no unified standard for measuring environmental regulations, and related research studies use the pollutant emission compliance rate or pollution control input costs [33, 34]. These approaches can partly reflect the intensity of regional environmental regulations, but they also suffer from endogeneity. Chen et al. [35] proposed a method to use the frequency of environment-related terms (i.e., PM_2.5_, PM_10_, CO_2_, SO_2_, air, pollution, ecology, green, emissions, energy consumption, low carbon, environmental protection, emissions reduction, and chemical oxygen demand) in government work reports to measure environmental regulations. This method has two advantages: First, environment-related terms cover a wider range that more comprehensively measures regional environmental management efforts. Second, government work reports are usually released at the beginning of the year, and the following economic activities do not have a reverse impact, which can mitigate endogenous problems to a certain extent. Due to these advantages, our study draws on this method.

#### 4.1.3. Moderator Variables

Officials' promotion incentives (Age) are one of the moderator variables. The level of government in China is positively correlated with the division of labor between the party committee and the government. Party secretaries have become the de-facto core of decision-making. An official's age is an essential factor for measuring promotion incentives. According to the retirement age limit of 60 years for the leading positions of prefecture-level municipalities, 55 years is generally a turning point for the strength of promotion incentives. Party secretaries are high-incentive officials if they are under 55 when they take office and low-incentive officials if they are 55 and older [36]. Following this logic, promotion incentives are characterized based on the party secretary's age when taking office, denoted as Age. Age is recorded as 1 when the party secretary takes office at an age less than 55 and 0 when it is greater than or equal to 55.

Officials' turnover (Turnover) is another moderator variable. According to the existing method, turnover is equal to 1 if replacement happens and 0 otherwise. If replacement happens before June 30, we set that year as turnover and the following year as otherwise.

#### 4.1.4. Control Variables

In addition to environmental regulations, other factors may also affect environmental improvement. We adopt the following control variables to eliminate the effects of noncritical factors [37]:

- City scale (CityScale): the reasonable city scale can reduce pollution emissions and improve environmental governance by enhancing the division of labor [38]. We use the total population of a municipal district as a proxy for the city scale.
- Technology level (Technology): the level of technology is an essential factor for determining pollutant emissions. It is expressed by the number of green invention patent applications in each city.
- Industrial structure (Industry): the secondary sector, specifically industry, is the principal source of pollutant emissions. The industrial structure is measured by the share of industrial value added in the city's GDP.
- Opening-up level (Open): the higher the level of openness in a region, the more deeply it can participate in the division of labor and absorb advanced external technology efficiently. We employ the actual amount of foreign investment used as a proxy for the opening-up level.
- Economic development (Economy): economic development and pollution are closely linked. We use the per capita GDP to measure a region's economic development level.

### 4.2. Data Source

The study manually collected the data on 276 cities from 2003 to 2019 based on availability. Relevant data were obtained from the Statistics Yearbooks of China 2004–2020, the Statistics Yearbooks of China City 2004–2020, government work reports, and the Database of the National Bureau. The information on party secretaries was available from the Database of China Local Party and Government Leaders. All indicators involving price factors were deflated to the year 2003 by the relevant price indices to weaken the influence of inflation factors on data fluctuations. The variables were treated with a logarithm to reduce the influence of fluctuation and heteroscedasticity with the exception of dummy variables.

### 4.3. Model Specification

To capture the moderating effect of promotion incentives on the effectiveness of environmental regulations, we constructed the following benchmark model with the example of wastewater emissions as

(1) $$\begin{array}{c} WaterI_{it}=\beta_{0}+\beta_{1}{ER}_{it}+\sum \beta_{j}CVs+\eta_{i}+\mu_{it}, \end{array}$$

where *i* and *t* denote the city and year, respectively. *β*_0_ is the constant term, and the coefficient of *β*_1_ indicates the impact of environmental regulations on environmental improvement. *β*_j_ denotes the regression coefficient for each control variable. Finally, *η*_i_ and *μ*_it_ represent the city effect and the random error term, respectively.

The moderator variables are centralized; subsequently, the interaction terms of environmental regulations with promotion incentives and officials' turnover are introduced based on the benchmark model, as shown in Equations (2) and (3). The coefficient of *α*_1_ in Equations (2) and (3) is the central interest as it indicates the moderating role of promotion incentives and officials' turnover. If the coefficient of the interaction term is significant, it suggests that moderating effects exist.

(2) $$\begin{array}{c} WaterI_{it}=\beta_{0}+\beta_{1}{ER}_{it}+\alpha_{1}\left({ER}_{it}*{Age}_{it}\right)+\alpha_{2}{Age}_{it}+\sum \beta_{j}CVs+\eta_{i}+\mu_{it}\text{,} \end{array}$$

(3) $$\begin{array}{c} WaterI_{it}=\beta_{0}+\beta_{1}{ER}_{it}+\alpha_{1}\left({ER}_{it}*{Turnover}_{it}\right)+\alpha_{2}{Turnover}_{it}+\sum \beta_{j}CVs+\eta_{i}+\mu_{it}\text{.} \end{array}$$

## 5. Empirical Results and Analysis

### 5.1. Summary Statistics

Table 1 reports the results of descriptive statistics for variables. The emissions of various pollutants and the level of environmental regulations vary greatly due to different stages of development.  Figure 2 depicts the age of party secretaries taking office and the corresponding number of secretaries. Findings show that the large number of party secretaries takes office at age 53, a total of 148, accounting for 11.41% of the total sample.  Figure 3 depicts the number of cities with party secretary turnovers, and a total of 1,296 turnovers occurred within the sample. The high-frequency years for party secretary changes are 2003, 2008, 2013, and 2017; these years correlate mainly to local transitions surrounding the Congress party.

### 5.2. Benchmark Regression and Robustness Tests

#### 5.2.1. Benchmark Regression Results

The covariance test is performed on the variables before regression analysis. The results show that the variance inflation factor values are all less than 10, so there is no multicollinearity among the variables.  Table 2 lists the benchmark regression results with the emission intensity of each pollutant as the dependent variable. It is found that the estimated coefficients of environmental regulations for each pollutant category are always negative and are all significant at the 1% level (*β*_1_ = −0.314, *p* < 0.01; *β*_1_ = −0.111, *p* < 0.01; *β*_1_ = −0.266, *p* < 0.01; *β*_1_ = −0.122, *p* < 0.01; *β*_1_ = −0.470, *p* < 0.01; and *β*_1_ = −0.157, *p* < 0.01, respectively); that is, environmental regulations effectively reduce the emission intensity of each pollutant. Environmental regulations have improved green production and resource utilization efficiency by encouraging enterprises to invest more in research so as to eliminate the backward production capacity. This is also consistent with the reality that China's environment has gradually improved in recent years. For the control variables, the estimated coefficients are generally consistent with expectations.

#### 5.2.2. Robustness Tests

Robustness tests are performed by reducing the endogeneity and replacing the dependent variables.

*(1)Endogeneity*. The explanatory variables are endogenous when correlated with the random perturbation term, which results in biased regression results. The omitted variables and reciprocal causality are important reasons for endogeneity. Individual fixed-effects models can be used for omitted variables to reduce the effect of unobservable factors, while the reciprocal causality problem needs to be solved with the instrumental variable (IV) approach. Environmental pollution could have a reverse effect on environmental regulations, mainly because the government may introduce more regulatory policies on environmental governance when the area suffers from pollution seriously. The choice of IV is highly artistic and creative. Since it is challenging to choose IV for environmental regulations, based on relevant research [39, 40], our study starts from the lagged term of endogenous variables. The lagged term of environmental regulations is highly correlated with current environmental regulations. In contrast, environmental pollution in the current period does not affect the level of previous environmental regulations, so the lagged term of environmental regulations initially satisfies the IV requirement. Therefore, this study chooses the one-period lag of environmental regulations as the IV. The benchmark regression is reanalyzed using two-stage least squares (2SLS), and the relevant results are listed in Table 3 The underidentification test and the weak IV test indicate that the IV is reasonable. Comparing the results in Table 2, the estimated coefficients of environmental regulations are all correspondingly higher (*β*_1_ = −0.281, *p* < 0.01; *β*_1_ = −0.477, *p* < 0.01; and *β*_1_ = −0.442, *p* < 0.01, respectively) after controlling endogeneity, indicating that the benchmark regressions mixed with endogeneity tend to underestimate the improvement effect of environmental regulations. In summary, after considering endogeneity, the direction and significance of the impact remain unchanged although the value fluctuates to some extent. Consequently, the benchmark regression results are robust and reliable on the whole.

*(2) Substitution of Dependent Variables*. By replacing the dependent variables in the benchmark regression from pollutant emission intensity to pollutant emissions, the corresponding regression results are reported in Table 4. The findings indicate that, except for slight fluctuations in the magnitude of the estimated coefficients, the effect of environmental regulations on all types of pollutants is still significantly negative (*β*_1_ = −0.155, *p* < 0.01; *β*_1_ = −0.081, *p* < 0.01; *β*_1_ = −0.107, *p* < 0.01; *β*_1_ = −0.091, *p* < 0.01; *β*_1_ = −0.348, *p* < 0.01; and *β*_1_ = −0.127, *p* < 0.01, respectively), indicating that environmental regulations do have a positive effect on reducing both the intensity of pollutant emissions and the total amount of pollutant emissions.

### 5.3. Moderating Effect Tests

#### 5.3.1. The Moderating Effect of Promotion Incentives

Theoretically, promotion incentives may have a moderating effect on the effectiveness of environmental regulations through GEC. To prove Hypothesis 1, we obtain the relevant regression results through Equation (2). To verify the robustness of the regression results, tenure is included in delineating the strength of promotion incentives. The study examined two scenarios that included 3-year tenure and 5-year tenure and one that did not include the year-by-year promotion incentive delineation criteria. Specifically, columns (2) and (3), columns (5) and (6), and columns (8) and (9) of Table 5 show that the coefficients of interaction terms in both soot and SO_2_ are positive and significant (*α*_1_ = 0.053, *p* < 0.05; *α*_1_ = 0.044, *p* < 0.05; *α*_1_ = 0.036, *p* < 0.01; *α*_1_ = 0.019, *p* < 0.05; *α*_1_ = 0.044, *p* < 0.01; and *α*_1_ = 0.038, *p* < 0.01, respectively). Promotion incentives have a positive moderating effect on the relationship between environmental regulations and air pollution. Since pollutant emission intensity is an inverse indicator, high promotion incentives weaken the effectiveness of environmental regulations for both categories of air pollutants in all three classification cases. In contrast, the positive moderating effect of promotion incentives is insignificant in wastewater and even shows a negative moderating effect (*α*_1_ = −0.012, *p* < 0.10) in the 5-year tenure criterion. Ulteriorly, it reveals that the distorting effect of promotion incentives on environmental regulations is more likely to occur in the area of air pollutants instead of water pollution from the perspective of GEC. Thus, Hypothesis 1 is partially verified because it does not consider pollutant heterogeneity.

The heterogeneity in the moderating effect of promotion incentives on different pollutants may be associated with the variation in pollutant spillover. Compared with wastewater, air pollutants have a substantial spillover. Especially in the research sample where prefecture-level cities dominate, the spillover is more significant due to the small area of jurisdiction. Moreover, air pollutants are more likely diluted and diffused by the wind. Therefore, the benefits and costs of air pollution control will be uncertain if relevant systems and collaborative governance mechanisms are not sound. Air pollutant emissions are prone to resulting in beggar-thy-neighbor situations and “race to the bottom” competitions. The spillover of wastewater is weak, and the boundary is clearly defined. With the implementation of the “river chief system,” the four-level river chief system (i.e., province, city, county, and township) in China has been established; the river chief system is also maintained by the key leaders of local governments. The river chief system adds political factors to water pollution control and promotes “yardstick competition” among regions. In the context of gradually increasing environmental performance appraisal, strengthening water pollution control can also give local officials a green label and increase promotion leverage to some extent.

To mitigate side effects caused by focusing on economic growth alone, the evaluation of officials has moved in a comprehensive and coordinated multidimensional direction. The central government has placed considerable value on green development since the 18th CPC National Congress in 2012, and the proportion of environmental indicators used in evaluating officials has also gradually increased. Therefore, taking 2012 as the node, we examine whether the moderating effect of promotion incentives changes by dividing the whole sample into two periods: 2003–2012 and 2013–2019. To save space, we only report the coefficients of interaction terms in the moderating effect model in Table 6 (we do the same in Tables 7 and 8). The comparison between the two different periods shows that the positive moderating effect of promotion incentives on air pollutants has increased numerically and significantly in varying degrees from 2013 to 2019, which implies that the official governance has not effectively reversed the trend of GEC in air pollutants. The moderating effect of promotion incentives on water pollution does not change significantly in the two periods, and neither period reaches statistical significance.

Although the environmental assessment indicators for officials are gradually increasing, it is awkward that the binding force is still limited. Environmental governance requires long-term investment and has a significant lag in effectiveness. It may be difficult to see the results of environmental governance within limited tenure, but it increases the performance of the next official. Therefore, local officials do not have sufficient incentives to invest in environmental governance. Furthermore, compared with the direct positive incentive of economic growth on officials' promotion, the current environmental appraisal is mainly in the form of “punishment,” which means that local officials will be held accountable only when major environmental accidents occur in their jurisdictions. We also notice that anticorruption efforts have increased unprecedentedly [41] and corruption behaviors have been effectively deterred since 2012. However, the empirical results do not show that promotion incentives have a weakened positive moderating effect on the effectiveness of environmental regulations. This is primarily because the concept of GEC used in this study contains not only corrupt collusion but also the complicity of local governments in allowing enterprises to adopt an unclean production mode for economic growth [42]. The latter, which accounts for the majority, is mainly caused by an extensive development concept without corruption and benefit exchange.

Significant differences exist between the city level and developmental stage among cities (municipalities, provincial capital cities, independent planning cities, and ordinary prefecture-level cities). Therefore, there should be heterogeneity in the moderating effect of promotion incentives among different city levels. The sample of 276 cities is divided into 243 ordinary prefecture-level cities (abbreviated as general cities) and 33 municipalities, provincial capital cities, and independent planning cities (abbreviated as high-level cities) to explore heterogeneity. The regression results for subsamples are presented in Table 7. Specifically, in the case of water pollution, columns (1), (4), and (7) show that the coefficients of the interaction terms are small and do not reach statistical significance in 243 general cities. In high-level cities, the coefficients are significantly negative (*α*_*1*_ = −0.044, *p* < 0.01 and *α*_*1*_ = −0.023, *p* < 0.10) in columns (4) and (7), except at the 3-year tenure criterion. In the case of soot, columns (2), (5), and (8) show that the coefficients of the interaction terms are significantly positive (*α*_1_ = 0.046, *p* < 0.05; *α*_1_ = 0.044, *p* < 0.01; and *α*_1_ = 0.052, *p* < 0.01, respectively) in general cities; in high-level cities, it is only significant at the 10% level (*α*_1_ = 0.105, *p* < 0.10) with the 3-year term criterion in column (2). In terms of SO_2_, the moderating effect of promotion incentives is not significantly different between general and high-level cities.

Overall, promotion incentives in high-level cities have a more substantial negative moderating effect and a weaker positive moderating effect on the relationship between environmental regulations and environmental pollution than in general cities. Several reasons can account for this phenomenon. On the one hand, high-level cities have more stringent environmental standards and higher public demand for the environment. Moreover, compared with general cities, high-level cities are already at a more advanced economic developmental stage and have a weaker motivation to develop the economy by destroying the environment. On the other hand, high-level cities experience a more robust legal system and vigorous public scrutiny, which increase the cost of collusion and the chances of exposure accordingly. As a result, high-level cities tend to be more cautious about collusion.

#### 5.3.2. The Moderating Effect of Officials' Turnover

Frequent turnover of principal local officials will disrupt the existing collusion network and create a sensitive deterrent period, thus restraining the behavior of all parties. As a result, officials' turnover may negatively moderate the relationship between environmental regulations and pollution, thereby contributing to environmental improvement. The relevant regression results shown in Table 9 are obtained by Equation (3) to test Hypothesis 2. Considering the lagged effect of officials' turnover, we take a one-period lag of officials' turnover. Moreover, according to Figure 3, the years (2003, 2008, 2013, and 2017) are the peak years for turnover, and the sample of these 4 years is excluded to reduce the impact of predictable turnover; corresponding results are shown in columns (4)–(6) of Table 9. From the full-sample regressions in columns (1)–(3), the findings show that similar to the moderating heterogeneity of promotion incentives, the moderating effect of officials' turnover is also significantly heterogeneous across pollutants. From the results presented in column (1), the coefficient of the interaction term in wastewater is negative and significant at the 5% level (*α*_1_ = −0.018,*p* < 0.05), indicating that officials' turnover has a negative moderating effect on the relationship between environmental regulations and water pollution. Consequently, it further suggests that officials' turnover has a deterrent effect on water pollution collusion, which will facilitate the effectiveness of environmental regulations. In the area of air pollutants, soot, and SO_2_, the moderating effect of officials' turnover is insignificant. Although the coefficient of the interaction term in SO_2_ is negative (*α*_1_ = −0.014), it does not reach statistical significance. After excluding the peak years of turnover, the significance of the estimated coefficients does not change compared to that of the whole sample, with only minor fluctuations in values.

Compared to wastewater, air pollutants have a high spillover and boundaries are more blurred. Even though officials' turnover can create shock damage to collusion, the deterrent effect on air pollutants is weak. Hypothesis 2 is also partially verified.

Following the idea that the moderating effect of promotion incentives is heterogeneous under different city levels, is there also city-rank heterogeneity in the moderating effect of officials' turnover? Therefore, based on the classification of the city rank mentioned above, this study examines differences in the moderating effects of officials' turnover under city-rank heterogeneity, and the results are presented in Table 8. Columns (1) and (3) show that the coefficients of the interaction terms are significantly negative (*α*_1_ = −0.025, *p* < 0.01 and *α*_1_ = −0.019, *p* < 0.10), which means that officials' turnover negatively moderates the intensity of wastewater and SO_2_ emissions in general cities. By contrast, only one coefficient of the interaction term is negative (*α*_1_ = −0.007) in the intensity of wastewater emissions in high-level cities in column (1), but it does not reach statistical significance. Moreover, from columns (4)–(6), after excluding the peak years of turnover, the direction of the moderating effect does not change, with only minor fluctuations in values and significance.

Compared with high-level cities, the collusion deterrent effect caused by officials' turnover is more significant in improving the effectiveness of environmental regulations in general cities. General cities still lag in terms of the development stage, legal environment, and government-enterprise relationship, and enterprises depend more on local governments. Therefore, the effect of fractured collusion networks caused by official mobility can be more profound in general cities.

## 6. Conclusions and Policy Recommendations

### 6.1. Conclusions

Environmental pollution limits the sustainability of economic development and significantly impacts the transmission capacity and pathogenicity of COVID-19. Therefore, effective environmental management will create a win-win situation for the ecological civilization and COVID-19 pandemic control. Based on the novel perspective of GEC, this study constructs a theoretical logic framework to explore the moderating effects of officials' promotion incentives and turnover on the effectiveness of environmental regulations using the balanced panel data from 276 cities in China from 2003 to 2019. To sum up, the main findings are as follows: First, environmental regulations do effectively restrain environmental pollution, including pollutant emission intensity and total emissions. Second, the positive moderating effect of promotion incentives on the effectiveness of environmental regulations is reflected in air pollutants but is not conspicuous in water pollution. In the new developmental stage (2013–2019), the binding force of the officials' environmental appraisal is still limited, so the moderating effect of promotion incentives remains predominantly positive. In terms of city-level heterogeneity, compared with general cities, promotion incentives in high-level cities have a weaker positive but a more potent negative moderating effect. Third, the collusive deterrent effect of officials' turnover negatively moderates the effectiveness of environmental regulations mainly in water pollution rather than air pollution. Compared with high-level cities, officials' turnover in general cities is more conducive to the effectiveness of environmental regulations.

### 6.2. Policy Recommendations

Strengthening pollution management and implementing green development are sufficient guarantees to coordinate COVID-19 controls and social development. The economic development model is the internal logic behind the moderating effects of promotion incentives and official turnover on the efficiency of environmental regulations. Transition economies represented by China have abundant labor resources but generally weaker social institutions and high transaction costs, so they rely on massive resource inputs to drive economic growth in the early developmental stages. GEC is the primary institutional driver of extensive development, which satisfies the parties' frenzied pursuit of economic growth in the short term. The extensive development model, characterized by high input, heavy pollution, and low efficiency, is unsustainable with the disappearing demographic dividend, tightening resource constraints, and rising transaction costs. Therefore, it is necessary to gradually improve the system construction, cut off the chain of GEC, and release the innovative vitality of enterprises to make the transformation into an intensive development model [43]. Otherwise, it is straightforward to fall into the middle-income trap. To break away from the sloppy development model, the following policy recommendations are also essential for transition economies with national conditions similar to those in China:

1. Scientific resumption of production: Owing to the severe economic impact of COVID-19, governments are prone to boosting the economy in the short term by relaxing regulatory policies, which may lead to a high incidence of GEC. Therefore, governments at all levels should firmly establish the concept of green development and scientifically organize the resumption of work and production; otherwise, the stimulation of the economy at the expense of the environment may lay a hidden danger for the spread of the COVID-19 virus.
2. Rethink the evaluation mechanism of officials: The evaluation mechanism determines the behavior of local officials. In addition to increasing the weight of environmental indicators, the central government should innovate and adjust officials' evaluation methods, which are invariably in the form of “punishment.” Dredging environmental pressure transmission can reverse local officials' one-sided pursuit of GDP and shape the official governance model of “growth for harmony.”
3. Accelerate the formation of regional joint governance mechanisms: For pollutants with a high spillover, the regional-coordinated governance mechanism can be formed by strengthening the vertical management of central-level or upper-level governments. The externality of pollution is gradually internalized to reduce the race to the bottom by forming a regional coordination governance mechanism.
4. Clarify the division of responsibilities: The “lifelong responsibility system for environmental damage” restrains wanton pollution behaviors under promotion incentives by setting policy red lines. However, the system still needs a more precise division of responsibilities and a perfect procedure to achieve realistic and lifelong responsibility.
5. Strengthen the legal system: While the officials' turnover may have a deterrent effect on collusion, new collusion networks can quickly emerge. Therefore, relying on the officials' turnover to improve the environment is not a long-term solution. A more sustainable plan is to improve the legal system and build a new type of proclear government-enterprise relationship.

### 6.3. Limitations and Future Research Directions

The limitations of this study point the way to future research, and three limitations stand out. First, the robustness of the empirical results can be further verified using additional measures of promotion incentives as well as mayoral data. In addition to the age factor, external factors such as GDP growth rates, fiscal surplus, and unemployment rates also measure promotion incentives in different dimensions. Mayors are an important faction that influences the regional economy, so the robustness of the results can be further tested by using multiple promotion incentive measures and combining them with mayoral data. Second, the impact of heterogeneity in the types of officials' turnover on collusion deterrence needs to be focused on. Officials' turnover includes retirement, promotion, reassignment, and corruption, which may cause differences in the damage degree of GEC. Therefore, future research studies should probe the impact of this variability by grouping or setting up dummy variables. Third, more pollutants need to be included in future research studies. Integrating data availability and workload, three representative pollutants (wastewater, soot, and SO_2_) were included in this study. Solid waste with lower spillover and nitrogen oxides in air pollutants can be introduced to further verify the robustness of the relevant results.

## Figures and Tables

**Figure 1:** Logical framework.

**Figure 2:** Age and frequency of party secretaries taking office.

**Figure 3:** Number of cities with party secretary turnovers.

**Table 1:** Descriptive statistics of the main variables.

Variable set	Variables	N	Mean	Sd	Min	Max
Dependent variables	WaterI (t/10^4^ yuan)	4692	30.907	50.761	1.181	2069.061
	Water (10^4^t)	4692	7132	9748	48	96501
	SootI (t/10^4^ yuan)	4692	0.017	0.046	0	1.535
	Soot (10^4^ t)	4692	2.916	7.770	0.004	325.726
	SO_2_I (t/10^4^ yuan)	4692	0.028	0.037	0	0.488
	SO_2_ (10^4^t)	4692	5.296	5.921	0.006	68.316

Independent variables	ER (number)	4692	25	15	1	110

Moderator variables	Age (0, 1)	4692	0.789	0.408	0	1
	Turnover (0, 1)	4692	0.277	0.447	0	1

Control variables	CityScale (10^4^p)	4692	145	193	14	3190
	Technology (number)	4416	280	1125	0	26435
	Industry (%)	4692	47.78	10.88	9	90.97
	Open (10^4^ yuan)	4692	479313	1186146	0	20478082
	Economy (10^4^ yuan/p)	4692	1.539	1.568	0.189	21.050

**Table 2:** Benchmark regression results of environmental regulations on environmental pollution.

Variables	(1)	(2)	(3)	(4)	(5)	(6)
	WaterI		SootI		SO_2_I	
ER	−0.314^*∗∗∗*^(−27.95)	−0.111^*∗∗∗*^ (−7.07)	−0.266^*∗∗∗*^ (−16.66)	−0.122^*∗∗∗*^ (−5.04)	−0.470^*∗∗∗*^ (−12.93)	−0.157^*∗∗∗*^ (−7.13)
CityScale		−0.008 (−0.31)		−0.007 (−0.16)		−0.208^*∗∗∗*^ (−5.35)
Technology		−0.172^*∗∗∗*^ (−22.26)		−0.093^*∗∗∗*^ (−7.88)		−0.355^*∗∗∗*^ (−32.67)
Industry		−0.108^*∗∗∗*^ (−3.04)		−0.055 (−1.01)		0.154^*∗∗∗*^ (3.08)
Open		−0.021^*∗∗∗*^ (−3.36)		−0.035^*∗∗∗*^ (−3.63)		−0.017^*∗∗*^ (−2.01)
Economy		−0.232^*∗∗∗*^ (−8.47)		−0.195^*∗∗∗*^ (−4.64)		−0.130^*∗∗∗*^ (−3.39)
Constant	−5.199^*∗∗∗*^ (−148.77)	−2.331^*∗∗∗*^ (−7.80)	−3.963^*∗∗∗*^ (−79.72)	−1.611^*∗∗∗*^ (−3.52)	−2.730^*∗∗∗*^ (−24.03)	−0.657 (−1.57)
N	4692	4692	4692	4692	4692	4692
*R * ^2^	0.150	0.277	0.059	0.075	0.082	0.406
City fixed	Yes	Yes	Yes	Yes	No	Yes

*Note.* The numbers in brackets stand for *t*-statistics;^*∗*^, ^*∗∗*^, and ^*∗∗∗*^ indicate significance at the level of 10%, 5%, and 1%, respectively, which are the same in the following tables except Table 3.

**Table 3:** IV-2SLS results.

Variables	(1)	(2)	(3)
	WaterI	SootI	SO_2_I
ER	−0.281^*∗∗∗*^ (−5.92)	−0.477^*∗∗∗*^ (−6.54)	−0.442^*∗∗∗*^ (−7.18)
Control variables	Yes	Yes	Yes
*N*	4692	4692	4692
*R * ^2^	0.255	0.023	0.380
City fixed	Yes	Yes	Yes
Kleibergen–Paap rk LM	269.455 (0.001)	269.455 (0.001)	269.455 (0.001)
Cragg–Donald Wald F	557.115	557.115	557.115

*Note.* The numbers in brackets stand for *z*-statistics; the numbers in the square bracket stand for *p* value; ^*∗*^, ^*∗∗*^, and ^*∗∗∗*^ indicate significance at the level of 10%, 5%, and 1%, respectively.

**Table 4:** Benchmark regression robustness test with replacement of dependent variables.

Variables	(1)	(2)	(3)	(4)	(5)	(6)
	Water		Soot		SO_2_	
ER	−0.155^*∗∗∗*^ (−14.08)	−0.081^*∗∗∗*^ (−5.14)	−0.107^*∗∗∗*^ (−6.69)	−0.091^*∗∗∗*^ (−3.72)	−0.348^*∗∗∗*^ (−20.21)	−0.127^*∗∗∗*^ (−5.51)
Constant	8.770^*∗∗∗*^ (256.18)	7.009^*∗∗∗*^ (23.44)	10.005^*∗∗∗*^ (200.63)	7.727^*∗∗∗*^ (16.65)	11.350^*∗∗∗*^ (211.97)	8.673^*∗∗∗*^ (19.83)
Control variables	No	Yes	No	Yes	No	Yes
*N*	4692	4692	4692	4692	4692	4692
*R * ^2^	0.043	0.195	0.010	0.044	0.084	0.348
City fixed	Yes	Yes	Yes	Yes	Yes	Yes

**Table 5:** The moderating effect of promotion incentives.

Variables	(1)	(2)	(3)	(4)	(5)	(6)	(7)	(8)	(9)
	3-year tenure criterion			5-year tenure criterion			Without considering tenure		
	WaterI	SootI	SO_2_I	WaterI	SootI	SO_2_I	WaterI	SootI	SO_2_I
ER	−0.099^*∗∗∗*^ (−4.88)	−0.172^*∗∗∗*^ (−5.50)	−0.198^*∗∗∗*^ (−6.95)	−0.076^*∗∗∗*^ (−3.10)	−0.225^*∗∗∗*^ (−6.01)	−0.212^*∗∗∗*^ (−6.20)	−0.111^*∗∗∗*^ (−5.26)	−0.220^*∗∗∗*^ (−6.84)	−0.244^*∗∗∗*^ (−8.27)
ER^*∗*^ Age	−0.013 (−0.94)	0.053^*∗∗*^ (2.53)	0.044^*∗∗*^ (2.29)	−0.012^*∗*^ (−1.90)	0.036^*∗∗∗*^ (3.61)	0.019^*∗∗*^ (2.11)	−0.001 (−0.02)	0.044^*∗∗∗*^ (4.63)	0.038^*∗∗∗*^ (4.43)
Age	−0.015 (−0.84)	0.004 (0.16)	0.035 (1.38)	−0.030 (−1.51)	−0.020 (−0.65)	0.026 (0.95)	0.007 (0.43)	0.065^*∗∗∗*^ (2.58)	0.042^*∗*^ (1.83)
Control variables	Yes	Yes	Yes	Yes	Yes	Yes	Yes	Yes	Yes
*N*	4692	4692	4692	4692	4692	4692	4692	4692	4692
*R * ^2^	0.277	0.077	0.407	0.278	0.078	0.407	0.277	0.083	0.410
City fixed	Yes	Yes	Yes	Yes	Yes	Yes	Yes	Yes	Yes

**Table 6:** The moderating effect of promotion incentives under different periods.

Variables	(1)	(2)	(3)	(4)	(5)	(6)	(7)	(8)	(9)
	3-year tenure criterion			5-year tenure criterion			Without considering tenure		
	WaterI	SootI	SO_2_I	WaterI	SootI	SO_2_I	WaterI	SootI	SO_2_I
2003–2012	−0.002 (−0.16)	0.005 (0.22)	−0.002 (−0.16)	−0.011 (−1.50)	0.029^*∗∗*^ (2.40)	0.009 (1.12)	−0.003 (−0.48)	0.021^*∗*^ (1.79)	0.012 (1.60)
2013–2019	−0.031 (−1.56)	0.041 (1.32)	0.071^*∗∗*^ (2.09)	0.001 (0.14)	0.048^*∗∗∗*^ (3.02)	0.055^*∗∗∗*^ (3.11)	0.007 (0.79)	0.039^*∗∗∗*^ (2.67)	0.048^*∗∗∗*^ (2.98)
Control variables	Yes	Yes	Yes	Yes	Yes	Yes	Yes	Yes	Yes
City fixed	Yes	Yes	Yes	Yes	Yes	Yes	Yes	Yes	Yes

**Table 7:** The moderating effect of promotion incentives under city heterogeneity.

Variables	(1)	(2)	(3)	(4)	(5)	(6)	(7)	(8)	(9)
	3-year tenure criterion			5-year tenure criterion			Without considering tenure		
	WaterI	SootI	SO_2_I	WaterI	SootI	SO_2_I	WaterI	SootI	SO_2_I
General cities	−0.007 (−0.54)	0.046^*∗∗*^ (2.05)	0.024 (1.22)	−0.005 (−0.75)	0.044^*∗∗∗*^ (3.99)	0.013 (1.42)	0.008 (1.22)	0.052^*∗∗∗*^ (5.16)	0.034^*∗∗∗*^ (3.82)
High-level cities	−0.029 (−0.96)	0.105^*∗*^ (1.86)	0.117^*∗∗*^ (2.38)	−0.044^*∗∗∗*^ (−3.24)	−0.010 (−0.42)	0.022 (0.98)	−0.023^*∗*^ (−1.69)	−0.004 (−0.18)	0.013 (0.62)
Control variables	Yes	Yes	Yes	Yes	Yes	Yes	Yes	Yes	Yes
City fixed	Yes	Yes	Yes	Yes	Yes	Yes	Yes	Yes	Yes

**Table 8:** The moderating effect of officials' turnover under city heterogeneity.

Variables	(1)	(2)	(3)	(4)	(5)	(6)
	Full sample			Sample excluding peak years of turnover		
	WaterI	SootI	SO_2_I	WaterI	SootI	SO_2_I
General cities	−0.025^*∗∗∗*^ (−3.28)	0.005 (0.50)	−0.019^*∗*^ (−1.85)	−0.018^*∗*^ (−1.96)	0.003 (0.27)	−0.023^*∗*^ (−1.80)
High-level cities	−0.007 (−0.51)	0.047^*∗*^ (1.66)	0.006 (0.24)	−0.008 (−0.40)	0.047 (1.42)	0.042 (1.29)
Control variables	Yes	Yes	Yes	Yes	Yes	Yes
City fixed	Yes	Yes	Yes	Yes	Yes	Yes

**Table 9:** The moderating effect of officials' turnover.

Variables	(1)	(2)	(3)	(4)	(5)	(6)
	Full sample			Sample excluding peak years of turnover		
	WaterI	SootI	SO_2_I	WaterI	SootI	SO_2_I
ER	−0.095^*∗∗∗*^ (−5.57)	−0.136^*∗∗∗*^ (−5.20)	−0.144^*∗∗∗*^ (−6.05)	−0.096^*∗∗∗*^ (−5.07)	−0.146^*∗∗∗*^ (−5.24)	−0.141^*∗∗∗*^ (−5.38)
ER^*∗*^ L.Turnover	−0.018^*∗∗*^ (−2.52)	0.015 (1.38)	−0.014 (−1.45)	−0.017^*∗∗*^ (−2.05)	0.009 (0.73)	−0.012 (−1.00)
L.Turnover	0.013 (0.83)	−0.054^*∗∗*^ (−2.22)	−0.054^*∗∗*^ (−2.42)	0.007 (0.38)	−0.054^*∗*^ (−1.90)	−0.074^*∗∗∗*^ (−2.78)
Control variables	Yes	Yes	Yes	Yes	Yes	Yes
*N*	4692	4692	4692	3588	3588	3588
*R * ^2^	0.278	0.077	0.407	0.267	0.093	0.391
City fixed	Yes	Yes	Yes	Yes	Yes	Yes

## Data Availability

The original contributions presented in the study are included in the article/supplementary material, and further inquiries can be directed to the corresponding authors.
